RETRACTED

# Extraction of Music Main Melody and Multi-Pitch Estimation Method Based on Support Vector Machine in Big Data Environment

**DOI:** 10.1155/2022/1074174

**Published:** 2022-08-31

**Authors:** Shaoru Liang, Ran Shu

**Affiliations:** ^1^School of Art, North University of China, Taiyuan 030051, China; ^2^Guizhou Normal College, Guiyang 550018, China

## Abstract

Main melody extraction and multi-pitch estimation are two important research topics in the MIR field. In this article, the SVM algorithm is used to analyze and discuss music melody extraction and multi-pitch estimation. In the part of multi-fundamental frequency extraction, this article first filters the song signal with equal loudness and weakens the energy of the high-frequency and low-frequency parts of the song signal. Thereafter, the multi-resolution short-time Fourier transform suitable for processing song signals is introduced. In addition, in order to avoid the sharp jump of the estimated melody pitch in the same note duration range, this article proposes a main melody extraction method combining the SVM algorithm with dynamic programming. In this article, more features are used to distinguish the pitch contour of vocal fundamental frequency from that of the nonvocal fundamental frequency, which does not only depend on energy or a certain feature. The experimental results show that the lowest octave error of this method is 1.46. Meanwhile, the recall rate of the algorithm can reach about 95%. This method not only improves the recall rate of the fundamental frequency of the human voice but also improves the recall rate and pitch accuracy rate of the whole main melody extraction system.

## 1. Introduction

As an effective carrier to express and convey emotions, the study of music is closer to people's lives. Although people are born with the ability to appreciate and identify music, it is very difficult for computers to analyze, understand, and retrieve music content [1]. Therefore, the research on MIR (music information retrieval) has been widely concerned by academic circles. The traditional music retrieval method is to match the song names or lyrics in the music retrieval library according to the entered keywords by the user, which is no longer in line with the needs of modern users. Users need a system that can not only satisfy the natural habit of listening to songs and recognizing songs but also improve the feedback and effect of retrieval [2]. Main melody extraction and multi-pitch estimation are important topics in the field of MIR. Main melody extraction, referred to as “melody extraction,” aims at automatically analyzing the audio content of a given piece of music by a computer and extracting the main melody of the piece of music [3]. The main melody extraction is mainly used in the humming retrieval system, and the main melody of songs is used as the retrieval feature. The definition of main melody extraction is to extract the main melody from a song signal and convert it into digital format features. Multi-pitch estimation is to estimate the pitch and number of notes in multi-tone music at each moment. The estimation of the pronunciation time and ending time of notes is sometimes included. Music is a kind of audio signal, so all the processing methods and retrieval methods of audio signals can be fully applied in the field of music analysis [4]. Extracting the main melody from the music signal is a technology that can help users directly interact with music by analyzing the information of audio files, and it is closely related to audio signal processing and MIR.

RETRACTED

The sum of the basic musical tones used in music is called the musical tone system. In the musical system, the smallest unit of pitch relation is a semitone, and the sum of two semitones is the whole tone. According to the types of music files, music melody extraction can be divided into two categories: melody extraction from MIDI files and melody extraction from audio files [5]. Each channel in the MIDI file stores the performance information of a musical instrument, so melody extraction is simple and the accuracy is high. The basic music information of MIDI includes sound symbols, dynamics, and time values. A symbol represents the pitch of a note. MIDI, a data format file based on musical notation symbols, stores music notes, instruments, rhythms, and other information in the file. Because the main melody of the song has been stored in the MIDI file, the main melody of the song can be obtained only by decoding the MIDI file. At present, music notation is a difficult problem in related fields. The main reason is that there will be a large number of overlapping harmonic components in each note that sounds at the same time, which will interfere with each other and hinder the recognition of each note. In addition, there are many kinds of music, different styles, various types of musical instruments, and various playing skills, so it is difficult to find a suitable general method to realize music notation. The primary element of musical works is music, and this waveform is periodic. Pitch, loudness, duration, and timbre are aspects of music that can only be experienced subjectively; however, each of these aspects has an objective counterpart. The estimation and analysis of each musical element, such as pitch, rhythm, melody, and others, is quite challenging, and at present, estimation errors are still quite large, while the error of the research findings on these elements is even higher [6]. In statistical learning, SVM (support vector machine) is a powerful machine learning algorithm. SVM was initially developed based on locating the ideal classification surface when the samples are linearly separable. Linear classifiers are the simplest and most efficient classifiers. We can see how an SVM is formed from a linear classifier. Finding an ideal classification hyperplane that satisfies the classification requirements, in order to ensure the classification accuracy and maximize the blank areas on both sides of the hyperplane, can be used to explain the basic concepts of SVM. The best classification of linearly separable data is theoretically possible with SVM [7]. The introduction of the kernel function changes the training samples from being linearly inseparable in low-dimensional space to being linearly separable in high-dimensional space. The analysis and discussion of music melody extraction and multi-pitch estimation are done in this article using the SVM algorithm. The article's innovations are as follows:

1. In this article, the statistical features of various music retrieval fields and logistic regression classifiers are used to introduce vocal frame judgment in the preprocessing stage so that the influence of nonvocal frames on the main melody judgment is reduced as much as possible, thus reducing the false alarm rate of main melody extraction and achieving the effect of improving the correct rate of the main melody in the system. The research shows that this method has high overall accuracy and low octave error rate.
2. The algorithm based on computational auditory scene analysis is used to realize singing separation and fundamental frequency extraction after preprocessing the input music signal. The main melody of the waveform file is also extracted at the same time as the fundamental frequency of the singing voice. Then, rather than relying solely on energy or a specific feature, the SVM model is used to distinguish between the pitch contour of the vocal fundamental frequency and that of the nonvocal fundamental frequency. This technique is suitable for songs with various signal-to-noise ratios and enhances the robustness of discrimination. It also performs well when handling songs with weak human voice signal-to-noise ratios.

RETRACTED

## 2. Related Works

Main melody extraction and multi-pitch estimation are two important research topics in the field of MIR, and many scholars have carried out in-depth research. Panda et al. improved a method originally used for the separation of harmonic percussion and used it for the separation of melodic accompaniment [8]. In the process of main melody track extraction, Fukayama and Goto focused on the MIDI music feature extraction before classification, the unbalanced situation of classification samples, and the reliability of classification results after two classifications so as to ensure the main melody track of MIDI music [9]. Calvo-Zaragoza and Oncina used SVM as a classifier to classify six different styles of music, namely pop music, classical instruments, piano music, folk songs, bel canto, and opera [10]. Chen et al. studied the theme judgment algorithm and proposed a theme judgment algorithm combining rules and statistical methods [1]. Langlois et al. believed that although the method for extracting pitches from monophonic music is not suitable for the simultaneous occurrence of multiple pitches, it is possible to combine the outputs of different methods to obtain a more credible result [11]. For the music to be processed, Zheng et al. extracted all its harmonic events and formed a set, each event in the set is a candidate for a fundamental frequency event, and then designed a support transfer algorithm to let these harmonic events vote each other to select the event with the highest support as the fundamental frequency [12]. The algorithm was tested on random chords synthesized from real instrument notes as well as computer-synthesized ensemble music, with promising results. Hsieh et al. chose a more effective main melody track extraction method to achieve the main melody extraction, that is, the SVM-based main melody track extraction method [13]. Kim et al.'s method is based on multi-fundamental frequency extraction of music, that is, it is considered that music is composed of the human voice and signals of various musical instruments. In order to obtain the fundamental frequency of human voice sources, it is necessary to extract candidate sound bases in the fundamental frequency domain, then use the short-term distinguishing features of vocal instruments to determine the main fundamental frequency to obtain the candidate acoustic fundamental frequency sequence, and, finally, use the long-term distinguishing characteristics of vocal instruments to determine the vocal frame to obtain a main melody fundamental frequency sequence [14]. Kroher et al. elaborated the main melody extraction method of the music library and the feature extraction and processing method of the humming feature including the fundamental frequency and the note and obtained the feature extraction effect through experiments. Finally, the humming retrieval system is tested from the system point of view, and the overall retrieval accuracy is obtained [15]. Baro et al. analyzed and compared the advantages and disadvantages of various multi-class classification methods and proposed a method combining prior knowledge and tree structure to construct a multi-classification system [16]. Correa et al. introduced the use of the harmonic scale feature description algorithm and implemented it and made a series of improvements to the harmonic scale feature description algorithm to make it suitable for multi-fundamental frequency extraction [17]. Chin et al. proposed an improved algorithm for high-volume audio tracks. The algorithm repeatedly deletes the musical instrument tracks that do not belong to the main melody according to certain rules and selects the audio track with the largest volume as the main melody track [18]. But since it ignores the main melody information that may be present in the lower voices, the description of the MIDI main melody is not accurate.

RETRACTED

Traditional methods have limited robustness, adaptability, and generalization ability, especially the characteristic parameters are mostly obtained by short-term stationary signal analysis. In this article, according to the actual situation, each music sample is preemphasized, framed, windowed, and muted. Then, the time and frequency domain perceptual features and pitch frequency features of the music sample are extracted to extract the matrix of the music sample and calculate the statistical features of the matrix. In addition, short-time Fourier transform and instantaneous frequency are used to estimate the sine of music mixed signal, and then the SVM algorithm is used to calculate melody pitch candidates. Finally, melody contour is obtained by the duration and continuity of pitch contour. The results show that, on the main melody extraction evaluation database, this method has high accuracy of main melody extraction, less false estimation, and its performance is improved. It also has good performance when dealing with songs with a low signal-to-noise ratio of human voice signals.

## 3. Methodology

### 3.1. Basic Music Theory Knowledge

Music is a way to express human thoughts and emotions. Music refers to an art composed of melody, rhythm, or harmony of human voices or musical instruments. The main melody is a musicological concept, which refers to the main phrases or musical forms that are reproduced or varied in the course of a musical work or movement. Generally speaking, polyphonic music has a main melody, accompanied by other notes. Melody is catchy, which is an important musical element for people to identify and remember music [19]. Melody recognition is to identify the main melody in a piece of music. Sound has three elements, namely pitch, loudness, and timbre. The vibration frequency of the sounding object determines the sound frequency, which is referred to as pitch. The pitch of an object increases with its vibration frequency. Loudness is a term used to describe the strength of sound, which is determined by the vibrating object's amplitude. The loudness of an object increases with its vibration amplitude. The subjective characteristics of sound that affect perception are referred to as timbre. The material, characteristics, and shape of the pronunciation body all play a role. The characteristic that distinguishes sounds is timbre. The perceptual characteristic of hearing known as pitch describes the order of sounds on a scale from low to high. Pitch measurement is subjective because it depends on the listener's subjective assessment. The fundamental frequency is an objective physical quantity, while pitch is a subjective perceptual one, but in the field of MIR, they are frequently treated equally. Signal shapes for sounds with the same pitch can vary. A single sine wave generates the simplest sound according to the number of frequency components. The sound currently only consists of the same frequency components as its pitch. A pure tone is the name for this type of sound. Polyphony is the term used to describe the sound created by superimposing multiple sine waves. The human ear perceives a sound as the same sound when its frequency is double that of another sound. However, the key is doubled and every time it is doubled, the human ear perceives a repetition. As a result, if a particular set of pitches is defined in one octave, those pitches can be used to represent those in other octaves. Therefore, people developed the Twelve Average Law, which establishes the pitch of each tone, in order to ascertain the absolute pitch of each tone in a musical tone. Twelve equally spaced semitones make up an octave, which is divided into twelve equal parts. The pitch is also established using this law.

RETRACTED

A chord is a sound effect produced by several notes arranged vertically according to certain rules. Chord recognition is to recognize the chord and its progression at every moment in polyphonic music. It can be seen as weakening the pitch estimation problem. The arrangement of each tone between two octaves is called “scale.” The mathematical calculation method of the precise pitch of each tone in the scale is called melody [20]. Besides having a fundamental frequency, human voices and musical instruments are accompanied by different harmonics and overtones. It is precisely because of these differences that different voices have different timbres. All the tones contained in a musical tone are called homophonic series. Music can be divided into single-part music and multi-part music. Single-part music has only one instrument or singing voice at a certain moment, so the typical pitch estimation method can be used to record the single-part music accurately. The sounds made by musical instruments are polyphonic, but they can be divided into harmony and disharmony. These characteristics are determined by the physical structure of the musical instrument. The so-called harmonic sound refers to the sound whose frequency components with significant energy are arranged at equal intervals. Each tone in the musical system is called the tone scale. And semitones are double in width, and a whole tone is the width of two semitones. Generally, in a sound, the energy at the pitch is the largest. While the frequency of the fundamental frequency is an integer multiple of the fundamental frequency, there will also be larger energy. This kind of frequency sound wave located at an integer multiple of the fundamental frequency is called harmonic. The melody of music embodies the main idea of music and is the soul of music. The characteristic of a singer's singing melody is that it is the continuity of a single note with different pitches in time, that is, there is only a single note at a certain moment. At present, it is urgent to solve the problem of multi-part music notation, that is, to identify each concurrent note at each moment from a piece of the music signal, form a score, and record it. Because this kind of music signal contains many notes which are concurrent according to the harmonic structure, and the spectrum overlap phenomenon is common, music notation is extremely challenging, and it is one of the difficult problems in the MIR field. Compared with polyphonic pitch estimation, melody recognition is easier. It only needs to detect one fundamental frequency at every moment, and this fundamental frequency is usually the most obvious. One application of melody recognition is audio-based retrieval, that is, the user provides a piece of music to the computer, and the computer recognizes its melody, and compares it with the melodies of other music in the database for retrieval.

### 3.2. SVM Algorithm

The binary classification issue was the initial target of SVM. The main goals of this approach are to maximize the classification interval while maintaining high classification accuracy, separate the two types of samples as accurately as possible, and find the best classification hyperplane in order to improve generalization ability. SVM is a very practical method that targets the issue of learning with small samples. It essentially only requires a small number of samples to perform effective machine learning, rather than a large number of samples. SVM's fundamental idea was developed from the ideal classification surface in the case of linear separable classes. The best classification surface is used to identify samples that fall into the two categories −1 and 1, and the points of these samples are farthest from the classification surface. Statistical learning theory and structural risk minimization serve as the theoretical foundation for SVM. The goal of this method, which was developed for use with small samples, is to strike a balance between generalization and model complexity so that the model is not overly complex, can make accurate predictions, and has good generalization capabilities. The principle of structural risk minimization is guaranteed because the higher the classification accuracy, the lower the empirical risk is, and the higher the maximum classification interval is, the lower the confidence risk is. SVM theoretically ensures that machine learning seeks the best solution because it eventually converts the machine learning problem into a quadratic programming problem. Since this is a convex quadratic programming problem, it can guarantee that the global optimal solution is sought, solving the non-global optimal solution issue with neural networks and other methods. The schematic diagram of the classification method is shown in Figure 1.

RETRACTED

When the data are linearly divisible, there must be two parallel hyperplanes. When the data are separated to the maximum extent, the edge data points will naturally fall on the plane, and the optimal classification plane is in the middle of these two parallel hyperplanes. For a linear classification problem, SVM directly constructs discriminant function in input space. The final SVM model only considers support vectors, and the number of support vectors is very small after screening, so its calculation speed is fast and the model is simple. Suppose there are *l* samples randomly and independently drawn from an unknown probability distribution function to form a training sample set:

(1) $$\begin{array}{c} \left\{\left(x_{i},y_{i}\right),i=1,2,3,\ldots ,l\right\}\;x_{i}\in R^{d}, \end{array}$$

where *y*_*i*_ ∈ {+1, −1} is the category identifier of the two types of samples. If *x*_*i*_ belongs to the first category, the output value is positive; if it belongs to the second category, the output value is negative. Therefore, the goal of learning is to construct a function to correctly divide as many samples as possible and maximize the classification interval, that is, the following optimization problem:

(2) $$\begin{array}{c} \underset{w,b,\xi }{\min}\frac{1}{2}w^{T}w+C\sum_{i=1}^{l}\xi_{i},\\ s.t.y_{i}\left(w^{T}x_{i}+b\right)\geq 1-\xi_{i},\\ \xi_{i}\geq 0,i=1,2,3,\ldots ,l, \end{array}$$

where *C* is the penalty parameter, and the larger the value, the greater the penalty for the classification error and the more emphasis is placed on the classification accuracy. In the process of structural risk minimization, two aspects should be considered comprehensively, which are empirical risk and confidence risk. From the empirical risk, it can be known that it represents the classification error of the classifier on a given sample, which reflects the learning ability of the classifier. The confidence risk represents the classifier's ability to classify unknown samples, so it is not an exact specific value, but a range of values, and it has a decisive influence on the whole generalization error.

RETRACTED

### 3.3. Music Melody Extraction and Multi-Pitch Estimation

Before extracting the features of music signals, in order to facilitate the analysis, each music signal must be preprocessed. It includes some steps, such as framing, windowing, preemphasizing, and distinguishing silent frames. These steps can be collectively referred to as short-time analysis preprocessing technology. According to whether the music contains singing or not, the main melody extraction methods can be divided into two categories: singing main melody extraction and general main melody extraction. If the music includes singing, the pitch sequence of singing is considered as the main melody; if there is no singing, the pitch sequence of the musical instrument with dominant energy will be the main melody. Due to the fixed frequency resolution, the low-frequency and high-frequency regions cannot meet the requirements at the same time when using a short-time Fourier transform to process music signals. Therefore, it is necessary to find a time-frequency transform method, so that the low-frequency region can meet the semitone-intensive characteristics and have a high-frequency resolution. The high-frequency region has rich dynamic characteristics and high time resolution. Because the waveforms of various sound source signals are mixed in the time domain, it is almost impossible to directly separate or detect the main melody, so it needs to be converted to other domains for analysis. This system selects the frequency domain commonly used by researchers and transforms the original music signal into the frequency domain for further analysis.

Music usually contains not only the sound signals of musical instruments but also the singing of human voices. This part of the letter can be directly understood as a speech signal. When processing the speech signal, we must consider the influence of nose and mouth radiation and glottic excitation on the power spectrum. There are relatively few components in the high-frequency part of music, and the frequency spectrum of the high-frequency part is difficult to obtain. Therefore, preemphasis must be introduced. The widely used preemphasis network is a first-order digital filter:

(3) $$\begin{array}{c} H\left(z\right)=1-\mu z^{-1}. \end{array}$$

The signal equation is:

(4) $$\begin{array}{c} y\left(n\right)=x\left(n\right)-\mu x\left(n-1\right), \end{array}$$

where *μ* is the preemphasis coefficient, which is a parameter close to 1. In this system, *μ* is taken as 0.97.  Figure 2 is a comparison diagram before and after preemphasis processing.

RETRACTED

The response curve of the equal loudness filter is approximately opposite to that of equal loudness filter. In this article, a 10-order infinite pulse corresponding filter is cascaded with a 2-order Butterworth high-pass filter. Through the function of two cascaded filters, the equal loudness curve is simulated, and the effect of equal loudness filtering is achieved. The music signal is a long-term nonstationary signal, but it can be regarded as a stable signal in a short time, and its characteristics are reflected in the short-term characteristics. Therefore, it needs to be framed and windowed. A piece of multi-part music can be expressed in the time domain as:

(5) $$\begin{array}{c} y\left(t\right)=x\left(t\right)+n\left(t\right), \end{array}$$

where *y*(*t*), *x*(*t*), and *n*(*t*) are the observation mixed signal, the main melody signal, and the additive accompaniment sound, respectively. Assuming that the single-tone signal is *x*(*i*), the autocorrelation function is defined as:

(6) $$\begin{array}{c} r_{t}\left(\tau \right)=\left(\frac{1}{W}\right)\sum_{j=t+1}^{t+w}x\left(j\right)x\left(j+\tau \right), \end{array}$$

where *τ* is called “hysteresis”; *t* is the moment of the current calculation; *W* is the size of the signal window participating in the calculation. This function achieves a maximum value at zero and a local maximum at the periodic point corresponding to the fundamental frequency and the periodic point corresponding to the harmonic frequency.

SVM can map the sample space to higher-dimensional space by kernel function when classifying samples, and for the samples themselves, they can also be high-dimensional feature attribute vectors. If we extract more independent feature attributes, the easier it is to separate classes from classes. The music features extracted in this article include MFCC combination, time domain features, frequency domain features, and gene frequency features. If zero padding is used in a short-time Fourier transform and the number of Fourier transform points is increased, the real frequency resolution will be smaller than the nominal frequency resolution. Reducing the frameshift can make the actual time resolution less than the nominal time resolution and increase the number of frames. The flow chart of music melody extraction and multi-pitch estimation method is shown in Figure 3.

RETRACTED

The main melody extraction system can be seen as a main melody pitch tracker. Its function is to calculate the value of the significance function *S*_*x*_(*f*_*τ*_, *τ*) within the possible range of the melody pitch frequency *f* at each time frame *τ* for a given input audio signal *y*(*t*). The function *S*_*x*_(*f*_*τ*_, *τ*) can be a time domain function or a frequency domain function, and the local estimation of the melody pitch is limited by the global timing constraints. Therefore, the melody pitch sequence value $\hat{f}$ is a vector that takes only one value per frame, namely:

(7) $$\begin{array}{c} \hat{f}=\text{arg}\underset{f}{\text{max}}\sum_{\tau }S_{x}\left(f_{\tau },\tau \right)+C\left(f\right), \end{array}$$

where *f*_*τ*_ is the *τ* element in *f*; *C*(*f*) stands for timing constraint.

Given a frame of music signal and the number of its notes, the pitch estimation of multi-tone can be regarded as a parameter estimation problem in the frequency domain, in which the complex spectrum is the observed data and the fundamental frequency is the parameter to be estimated. Assuming that the number of notes is *N*, then we can build a maximum likelihood model:

(8) $$\begin{array}{c} \left({\hat{f}}_{0}^{1},\ldots ,{\hat{f}}_{0}^{N}\right)=\arg\underset{f_{0}^{1},\ldots ,f_{0}^{N}\in F}{\text{max}}p\left(O|f_{0}^{1},\ldots ,f_{0}^{N}\right), \end{array}$$

where *O* represents the observed spectrum, *f*_0_^1^,…, *f*_0_^*N*^ is the fundamental frequency in *N* logarithmic scales, and *F* is the possible frequency range of the fundamental frequency. In this article, both frequency and amplitude are on a logarithmic scale, and the units are MIDI counts and dB, respectively.

When classifying samples, we can map the sample space to higher-dimensional space by kernel function, and for the samples themselves, they can also be high-dimensional feature vectors. In the sine extraction part, the frequency and amplitude of the music signal are detected and estimated to obtain the frequency spectrum of the signal. The saliency function part extracts the sine component in the frequency spectrum and calculates the saliency function. Pitch contour extraction part constructs the pitch contour line by saliency function. In the melody selection part, human voice detection and other errors such as octave errors are detected and corrected. Finally, the fundamental frequency sequence of the main melody is obtained. This article highlights and smooths the peak point and influences the frequency and amplitude of the peak point as little as possible. The purpose of this is to minimize the inaccuracy of the frequency value and amplitude value of the peak point caused by the digital signal processing in the time-frequency transformation process. The purpose of introducing preemphasis in this article is to relatively improve the components of the high-frequency part so that the frequency spectrum of the signal becomes very flat and the whole frequency band from high frequency to low frequency can be calculated with the same signal-to-noise ratio, which is convenient for spectrum analysis or channel parameter analysis.

RETRACTED

## 4. Result Analysis and Discussion

The sample categories of this article are divided into six different styles of music, namely pop music, piano music, classical music, bel canto, folk songs, and operas. Both training samples and test samples are selected artificially, and as training samples, their categories belong to prior knowledge. That is, the training process of the SVM classifier is based on the fact that the categories of training samples are known, and the two-class classification of SVM is to select the support samples that can best reflect the differences between the classes from the two classes of the known categories. In this experiment, a piece of music with a time length of about 10s is selected from the experimental data set as the research data so as to analyze and introduce the experimental results in detail. The function of time-frequency change is to get the candidate's fundamental frequency in the peak of the frequency domain, which is convenient for judging the candidate's fundamental frequency to get the fundamental frequency of the human voice. Therefore, one of the evaluation indexes of time-frequency change is the recall rate of the fundamental frequency of the human voice. In addition, in the classical music melody extraction system, the most important feature of the vocal fundamental frequency judgment is the frequency point energy, so the greater the frequency point fundamental frequency energy, the greater the probability of being judged as vocal fundamental frequency. The interval relationship between each subharmonic frequency and the fundamental frequency is shown in Table 1.

The sampling rate of training and testing data in this article is 44.1 kHz. The frame length and frame hop are 93 ms and 46 ms, respectively. During training, all frames of each sample are used to detect and collect peaks and harmonics. It is not necessary to deal with the song completely to reflect the category of music. Often, the style of a song only needs one or two fragments to fully explain its characteristics. Therefore, after selecting the correct music, it is necessary to intercept each piece of music. The unified input format of these music clips is .wav. The spectrogram of musical instrument components obtained after preprocessing in this article is different from the spectrogram of the original music signal. Because of its quasi-periodicity and short-term stability, the singing voice is still smooth along the time direction in a short time in the spectrogram. At the same time, due to the existence of accompaniment music produced by percussion instruments, it is smooth along the frequency direction in some time periods in the spectrogram. The results of sound bureau estimation in the presence of fundamental frequency are shown in Figure 4.

RETRACTED

Figure 4 shows that as the degree of detuning increases, the accuracy of treble estimation declines. The sensitivity of the two methods to fundamental frequency and harmonic frequency offset is similar, while the original pitch accuracy of the proposed method is marginally better than that of the KD method. When separating singing, the time-frequency unit is marked in accordance with the singing's fundamental frequency extraction results after the signal combination is complete. In this article, only the peak points are selected for energy mapping, which can not only ensure the superposition of the energy points of higher harmonics to the fundamental frequency but also eliminate the influence of the whole spectrum compressing the energy of other points. It will not cause the influence of “redundant energy” near the fundamental frequency in the subharmonic superposition algorithm. The experimental results of the recall rate of speech frames of different classifiers are shown in Figure 5.

The combination of various spectral peak pairs will make the improved Euclidean algorithm estimate the pitch value with octave error, and it will be retained as a candidate pitch because of its larger significance value. Methods using these pitches with octave errors to supplement the gap of pitch contour are proposed.  Figure 6 shows the original pitch accuracy of this method on different databases.

According to the statistical analysis results in Figure 6, the contour supplement strategy is helpful to improve the average original pitch accuracy of each database. Although the vocal tract has several resonance peaks, the sound energy will be concentrated in the following when the vocal portion of the music signal is voiced because the glottic excitation and the radiation from the nose and mouth will cause a high-frequency drop in the frequency spectrum. Since the majority of the energy is concentrated in the high-frequency region when voicing unvoiced sound, the short-time average zero-crossing rate can be used to separate voiced from unvoiced sound as well as to separate the voice signal from background noise. It can be used to determine where voiced and silent segments begin and end. The error situation of different algorithms is shown in Figure 7.

RETRACTED

The harmonic richness of speech is similar to that of musical sounds. Because the spectrum energy of speech is mainly concentrated in low frequency, it has fewer harmonic components than musical sounds. When the voice signal is mixed with the musical sound signal, its spectrum is similar to that of the musical sound, so it has a larger spectrum centroid than the voice itself.  Table 2 shows the performance comparison on different databases.

Experiments show that the proposed melody extraction method can extract the main melody from music audio. There is little difference, which indicates that the error rate of the proposed method is low. Moreover, this method can make use of more high-frequency components and will not suffer from the problem of insufficient resolution of spectral compression in the process of superposition of subharmonics.

## 5. Conclusions

For the purposes of understanding music, creating music, and automatically composing music, music content analysis has significant theoretical significance and practical application value. Two crucial components of music content analysis are main melody extraction and multi-pitch estimation, but when the music content is complex, these two issues have not yet been adequately resolved. SVM can resolve not only linear classification issues but also nonlinear and incomplete classification issues. It is possible to obtain a linear solution by using the hyperplane method to convert the nonlinear classification problem into a linear classification problem in a high-dimensional space. In addition, SVM has some fault tolerance and penalty parameters. The SVM algorithm is used in this article to analyze and discuss melody extraction and multi-pitch estimation in music. The main melody judgment algorithm suggested in this article filters out a significant portion of obvious pitch contours of the nonvocal fundamental frequency as a method to reduce their interference. Then, rather than relying solely on energy or a specific feature, the SVM model is used to distinguish between the pitch contour of the vocal fundamental frequency and that of the nonvocal fundamental frequency. According to the experimental findings, this method's lowest octave error is 1.46, and its recall rate can be as high as 95%. This demonstrates the low error rate and general reliability of the suggested method. This technique is suitable for songs with various signal-to-noise ratios and enhances the robustness of discrimination. It also performs well when handling songs with weak human voice signal-to-noise ratios. Even though this article produced some research findings, there is still some research to be done. To lower the ratio of missed detection and false alarm pitch and further increase the accuracy of multi-pitch estimation, it will be necessary to study various note combination rules and incorporate them into the algorithm.

RETRACTED

## Figures and Tables

**Figure 1:** Schematic diagram of the classification.

**Figure 2:** Comparison before and after preemphasis processing.

**Figure 3:** Method flow of music melody extraction and multi-pitch estimation.

**Figure 4:** Fundamental frequency or harmonic offset.

**Figure 5:** Experimental results of recall rate of speech frames with different classifiers.

**Figure 6:** The original pitch accuracy of this method on different databases.

**Figure 7:** Errors of different algorithms.

**Table 1:** Interval relationship between harmonic frequency and fundamental frequency.

Harmonic frequency	Frequency	Interval
2	2*f*_0_	Pure octave
3	3*f*_0_	Pure octave + pure fifth degree
4	4*f*_0_	Two octaves
5	5*f*_0_	Two octaves + major third
6	6*f*_0_	Two octaves + pure five degrees
7	7*f*_0_	Two octaves + pure seven degrees

**Table 2:** Performance comparison on different databases.

Database	Method	RPA (%)	RCA (%)	Octave error
ISMIR2004	MEA method	64.76	69.91	4.96
	Methods of this article	87.84	88.17	2.97

MIREX05 train	MEA method	65.11	68.85	3.64
	Methods of this article	86.79	86.91	1.46

MIR-IK	MEA method	61.37	65.34	6.58
	Methods of this article	89.74	87.05	3.64

## Data Availability

The data that support the findings of this study are available from the corresponding author upon request.
